RETRACTED

# The Clinical Efficacy and Economic Benefits of Recombinant Human Thrombopoietin for the Treatment of Chemotherapy or Chemoradiotherapy-Induced Thrombocytopenia

**DOI:** 10.1155/2022/2256690

**Published:** 2022-07-14

**Authors:** Wenxian Wang, Xiaodong Gu, Lan Shao, Zhiyong Shi, Guangyuan Lou, Zhengbo Song, Yiping Zhang

**Affiliations:** ^1^Department of Medical Oncology, The Cancer Hospital of the University of Chinese Academy of Sciences (Zhejiang Cancer Hospital), Hangzhou 310000, China; ^2^Institute of Basic Medicine and Cancer (IBMC), Chinese Academy of Sciences, Hangzhou 310000, China

## Abstract

Even though cytopenia caused by either chemotherapy or radiotherapy is a common complication in cancer patients, chemoradiotherapy remains an essential treatment for the majority of patients. The purpose of this study was to look into the clinical efficacy and cost-effectiveness of recombinant human thrombopoietin (rhTPO) in treating chemo- or chemoradiotherapy-induced grade II, III, and IV thrombocytopenia. From December 2019 to November 2020, 233 lung cancer patients admitted to our hospital with chemotherapy- or chemoradiotherapy-induced thrombocytopenia were enrolled and treated with rhTPO. The study's findings revealed a significant disparity in the use of concurrent chemoradiotherapy in patients with grade II, III, and IV thrombocytopenia. All costs, including rhTPO treatment costs, platelet costs, drug costs, and nondrug costs, tended to rise as the severity of thrombocytopenia increased. In the treatment of chemotherapy or radiotherapy-induced thrombocytopenia, rhTPO has shown good clinical efficacy. In the treatment of grade II thrombocytopenia, rhTPO has a favorable economic evaluation. As a result, early intervention and thrombocytopenia treatment should be provided, which warrants further clinical investigation.

## 1. Introduction

Thrombocytopenia is a hematologic disorder characterized by a low platelet count (<150 × 10^3^ cells/*μ*L blood) and is often a multifactorial disease. Platelets play an important role in the physiological system of the body, especially in the vascular injury response. Platelets prevent excessive blood loss after injury by forming a structural plug. Various receptors are present in the embolic layers of collagen, ADP, vascular septate von Willebrand factor, and fibrinogen. Major causes of thrombocytopenia include increased destruction, splenic sequestration and decreased platelet production by the bone marrow. The causative agents have been implicated in several types of thrombocytopenia, such as drug-induced thrombocytopenia, idiopathic thrombocytopenic purpura, HIV-induced, dengue, cirrhosis, leukemia, chikungunya, hepatitis C virus, malaria, and various infections. The incidence of thrombocytopenia in adults is 3.3 per 100000 per year, and the prevalence is 9.5 per 100000 adults.

RETRACTED

After receiving chemotherapy or chemoradiotherapy treatments, the patients with malignant tumors often suffer different grades of thrombocytopenia. More seriously, some of them even have bleeding tendencies, such as cutaneous, visceral, and intracranial hemorrhages which can lead to death in severe cases. Thus, prevention and treatment have become relatively difficult. Thrombocytopenia can alter the treatment course with chemotherapy or chemoradiotherapy, leading to a reduction in their doses or a delay of the next treatment cycle, or even treatment discontinuation, thus affecting the expected therapeutic effect [1, 2]. Due to functional inhibition of the bone marrow produced by chemotherapy or chemoradiotherapy drugs, chemotherapy- or chemoradiotherapy-induced thrombocytopenia result in the death and inhibition of megakaryocytes [3]. The clinical treatment of thrombocytopenia is very limited, such as reducing the dose of chemotherapy or chemoradiotherapy drugs, delaying chemotherapy or chemoradiotherapy, performing platelet transfusion, and administering recombinant human interleukin-11 (rhIL-11) and recombinant human thrombopoietin (rhTPO).

Platelet transfusion is one of the most direct treatments, it allows to rapidly increase the platelet level in patients undergoing chemotherapy or chemoradiotherapy. However, it usually causes several adverse reactions. In addition, platelets have a short lifespan and are difficult to collect and preserve. Repeated platelet transfusions lead to the development of antibodies and the destruction of transfused platelets, which affect the therapeutic efficacy [4–6]. Thrombopoietin, as a hematopoietic growth factor, is a thrombopoietin factor that stimulates hematopoietic stem cell proliferation and differentiation and regulates the proliferation, differentiation, maturation, and division of megakaryocytes to form functional platelets [7–9]. Recombinant human thrombopoietin is a full-length glycosylated TPO expressed by Chinese hamster ovary (CHO) cells using gene recombination technology followed by purification, which exhibits similar pharmacological effects as endogenous TPO in increasing platelet levels. The incidence of lung cancer in China is parabolically increasing with the aging of the population, urbanization of rural areas, aggravation of the urban industrialization process, serious pollution and destruction of the living environment, as well as the promotion of unhealthy lifestyles, especially the increasing number of smokers in China year after year. According to the latest data, lung cancer has become the most important type of cancer in China ranking No. 1. Its incidence and mortality are increasing rapidly and it is also one of the malignant tumors with the worst prognosis [10]. For this reason, more and more attention and urgency are being given to treatments relevant to lung cancer. Even though we have already entered the era of targeted therapy and immunotherapy, taking into account the economic cost, patient wishes, and other factors, chemotherapy or chemoradiotherapy are still indispensable treatments. Although chemotherapy- or chemoradiotherapy-induced thrombocytopenia constitutes a common complication in cancer patients, the clinical efficacy and economics of rhTPO in the treatment of grade II, III, and IV thrombocytopenia induced by chemotherapy or chemoradiotherapy in patients with lung cancer should be investigated in-depth.

RETRACTED

The pathogenesis of thrombocytopenia is currently thought to be due to the in vivo production of antiplatelet antibodies that cause excessive platelet destruction and a shortened platelet lifespan, whereas megakaryocytes in the bone marrow are normal or increased and megakaryocytes are degenerated and naive because the pathogenesis is related to autoimmunity. This condition is an acquired bleeding disorder. Etiological aspects of the disease, rubella, measles, chickenpox, mumps, infectious mononucleosis, and live viral injections, among others, have been identified. In recent years, experiments have confirmed that certain viruses, such as the varicella virus, can be the acute ITP etiology. The pathogenesis of chronic thrombocytopenia is that the antiplatelet antibody IgG (PAIgG), mainly produced by the spleen, binds specifically to the associated antigen on the platelet membrane through its Fab fragment, exposes the Fc fragment and binds to the Fc receptor of the giant cell, causing the platelet to be phagocytosed and destroyed; in addition, immune complexes (CICS) bind to Fc receptors on platelets via Fc fragments on their IgG molecules and activate complement C3, allowing C3 to be immobilized on platelets and finally recognized and phagocytosed by macrophages. The role of cellular immunity in this disease is unknown, with a known dysregulation of the proportion of helper and suppressor T cells and defective TA cell function. The major sites of platelet destruction are the spleen, liver, and bone.

Chemotherapy- or chemoradiotherapy-induced thrombocytopenia is frequently caused by the myelosuppressive side effect of antitumor therapy drugs, especially in megakaryocytes, resulting in a platelet concentration decreased in the peripheral blood. A platelet count below 50 × 10^9^/L can trigger mucosal or cutaneous hemorrhages, resulting in spontaneous bleeding as the platelet count continues to decline [11, 12]. At present, the pathogenesis of thrombocytopenia has not been fully clarified and most scholars believe that it is caused by excessive T cell-mediated platelet destruction, impaired megakaryocytopoiesis, and thrombopoiesis and a disturbed T-helper-cell (Th) balance [13].

RETRACTED

The lung is a hematopoietic organ. In animals, more than half of PLTs come from the lung, where megakaryocytes and a wide variety of hematopoietic progenitor cells are stored. These cells can be used to restore the hematopoietic capacity of damaged bone marrow. The blood vessels in the lung are narrower and therefore the resulting pressure is more conducive to the production of PLTs, or it may also happen that the lung releases a signaling molecule, which is more conducive to the production of PLTs from megakaryocytes [14]. For this reason, patients with lung cancer may have a low tolerance level to chemotherapy or chemoradiotherapy. In addition, some drugs in chemotherapy regimens have a greater impact on platelet count, e.g., carboplatin significantly inhibits PLT production and gemcitabine affects peripheral blood PLTs by influencing the maturation and differentiation of megakaryocytes; patients also often require multiple chemotherapy or chemoradiotherapy, so bone marrow suppression is more likely to occur; especially in patients receiving a wide range of complete lung radiotherapy, there is an aggravation of suppression in the bone marrow, producing grade III and IV thrombocytopenia and even causing bleeding from important organs [15]. Therefore, chemotherapy- or chemoradiotherapy-induced thrombocytopenia may pose a greater threat to the safety and life of lung cancer patients and for this reason, diagnosis and treatment should be made in time once it is found [16, 17]. rhTPO is a highly specific regulator of megakaryocyte growth and differentiation, which produces distinctive biological effects by binding to the specific MPL receptor, regulates the entire differentiation and maturation process of megakaryocytes, and promotes platelet production. rhTPO can act over a longer period with a half-life of approximately 40 h, reducing the requirements for platelet transfusion with a high level of tolerability and safety [18]. Previous studies have shown that rhTPO not only increases the number of platelets but also increases the mean platelet count at the trough level, shortens the duration of low platelet level, and significantly reduces the number of platelet transfusions [19]. As is well known, platelet transfusion is a common treatment for chemotherapy- or chemoradiotherapy-induced thrombocytopenia, but it may increase the risk of infectious diseases, produce transfusion reactions, and graft-versus-host disease (GVHD). In addition, platelet transfusion is relatively expensive and easily leads to a heavy economic burden on patients and their families. Therefore, the rhTPO can accelerate platelet recovery while compensating for the disadvantages of platelet transfusion [20, 21].

RETRACTED

Two drugs, recombinant human thrombopoietin (rhTPO) and recombinant human interleukin-11 (rhIL-11) have been approved by the National Medical Products Administration (NMPA) for the treatment of chemotherapy- or chemoradiotherapy-induced thrombocytopenia. Both can directly stimulate and induce megakaryocyte differentiation and maturation and promote thrombopoiesis, but rhTPO is more effective than rhIL-11 in regulating the early hematopoietic system [22]. In the meta-analysis of rhTPO for the treatment of chemotherapy-induced thrombocytopenia in malignant tumors reported by Cheng Han *et al.* [6], 34 randomized controlled studies involving a total of 2186 patients were included, and the results suggested that rhTPO was superior to rhIL-11 at increasing the highest platelet count, shortening the duration of thrombocytopenia, and reducing the incidence of adverse reactions and the proportion of platelet transfusion. In addition, according to the *Consensus on Clinical Diagnosis, Treatment and Prevention Management of Chemotherapy-induced Thrombocytopenia in China* (2018), when 10 × 10^9^/L＜PLT＜75 × 10^9^/L, medication should be applied [9]. However, there is no clear definition and description of when to start treatment, and the efficacy and economic differences at different treatment times are unknown. Thus, we aim to provide preliminary information about the efficacy and economics of rhTPO application in grade II, III, and IV thrombocytopenia.

The results of the study revealed that there are significant differences in whether or not concurrent chemoradiotherapy is used in patients with grade II, III, and IV thrombocytopenia. Further pairwise comparisons found that the difference in concurrent chemoradiotherapy between patients with grade II and III thrombocytopenia was statistically significant, suggesting that more attention should be paid to the changes in platelet count in those patients receiving concurrent chemoradiotherapy and therefore early intervention should be performed because those who receive thoracic radiotherapy may have a low tolerance level and it is not conducive to platelet production. As the severity of thrombocytopenia increased, the days of rhTPO treatment, the proportion of patients requiring platelet transfusion, time of increased platelets, delay of the next chemoradiotherapy cycle, and prolonged hospitalization due to platelet decline also increased. Further pairwise comparisons between patients with grade II, III, and IV thrombocytopenia indicated that the days of rhTPO treatment, the proportion of patients requiring platelet transfusion, time to increased platelets, delay of the next chemoradiotherapy cycle, and prolonged hospitalization due to platelet decline are all the minimum in patients with grade II thrombocytopenia. In addition, when it comes to the selection of therapeutic drugs or treatment regimens, not only the safety and efficacy of drug therapy but also economic factors should be considered, so that patients can obtain the best effect with the least economic burden while improving the effective utilization and allocation of pharmacological resources. The study also showed that with the increase in the severity of thrombocytopenia, the corresponding hospitalization costs also increased. The same trend is also observed in all in costs, rhTPO treatment costs, platelet costs, drug costs, and nondrug costs. All costs of the patients with grade II thrombocytopenia are the lowest. It is consistent with the results obtained from the above efficacy indicators. Also, it suggests that the application of rhTPO is more favorable when grade II thrombocytopenia occurs. In promoting the recovery of platelet levels, early use of rhTPO can provide more help for patients, to obtain more cost-effective treatment. Theoretically, by quickly solving the problem of thrombocytopenia, the treatment delay and dropout existing in severe thrombocytopenia are avoided, allowing to indirectly ensure a benefit for patients due to the adequate dose and cycle of chemotherapy or chemoradiotherapy. Since the followup duration is still short, the patient's long-term survival and prognosis cannot be investigated. In addition, it is difficult to distinguish whether adverse reactions that occurred in patients were caused by chemotherapy or platelet-stimulating drugs in the retrospective analysis of cases, so only drug costs within the direct medical costs are included in the cost measurement, while the costs produced by adverse drug reactions are not considered, which can also have an impact on the results of the pharmacoeconomic evaluation.

RETRACTED

## 2. Materials and Methods

### 2.1. General Information

A total of 233 lung cancer patients (179 males and 54 females, with an age range between 26 and 79 years and a mean of 61.94 ± 7.87 years) with chemotherapy- or chemoradiotherapy-induced thrombocytopenia were admitted and treated at our hospital in December 2019 to November 2020 were selected. Ninety-two (92) of the 233 patients received concurrent chemoradiotherapy and 141 patients did not; they have 1–16 (mean 6.19 ± 1.27) months of tumor history and a thrombocytopenic duration of 1–21 (mean 5.13 ± 0.62) days. According to the staging criteria of the Union for International Cancer Control, 45 patients were in stage I, 79 patients in stage II, 68 patients in stage III, and 41 patients in stage IV. A total of 100 patients had grade II thrombocytopenia, 94 patients had grade III and 39 patients had grade IV thrombocytopenia. Inclusion criteria: (1) patients with an expected survival >3 months; (2) patients >18 years of age; (3) patients with platelet count (PLT) less than 75 × 10^9^/L; (4) patients with normal bone marrow reserves; (5) patients with performance status score ≤2. Exclusion criteria: (1) patients with significant heart, liver, kidney, or other organ diseases; (2) pregnant or lactating patients; (3). patients predisposed to infections; (4) patients with disseminated intravascular coagulation; (5) patients with second primary tumor. This study has been reviewed and approved by the Ethics Committee of our hospital.

### 2.2. Study Method

Corresponding chemotherapy or chemoradiotherapy regimens were used in lung cancer patients by NCCN guidelines. After chemotherapy, if PLT was less than 75 × 10^9^/L, PLT was less than 50 × 10^9^/L and PLT was less than 25 × 10^9^/L, a dose of 15000U of rhTPO was injected subcutaneously once a day, and if PLT reached 100 × 10^9^/L or increased 50 × 10^9^/L than before rhTPO treatment, rhTPO was discontinued. rhTPO was used continuously for up to 2 weeks. Baseline conditions in patients with grade II, III, and IV thrombocytopenia, including gender, age, and concurrent chemoradiotherapy were compared. Differences in the days of rhTPO treatment, time to increased platelets after treatment, delay of the next chemoradiotherapy cycle, prolonged hospitalization due to platelet decline, increased hospitalization costs due to platelet decline, and with or without platelet transfusion of grade II, III, and IV thrombocytopenia were compared. Then, the pairwise comparisons of the aforementioned indicators were performed between patients with grade II, III, and IV thrombocytopenia.

### 2.3. Grading of Thrombocytopenia

According to the WHO grading system for thrombocytopenia, grade II thrombocytopenia corresponds to a platelet count between 50 × 10^9^/L and 75 × 10^9^/L; grade III thrombocytopenia corresponds to a platelet count between 25 × 10^9^/L and 50 × 10^9^/L, and grade IV thrombocytopenia corresponds to a platelet count of <25 × 10^9^/L.

### 2.4. Statistical Methods

In the data processing and analysis, the statistical software SPSS 22.0 was used. If the measurement data followed the normal distribution, they would be expressed as mean ± standard deviation, and the differences among the three groups were compared using analysis of variance (ANOVA). Otherwise, they were expressed as median and upper-lower quartiles; meanwhile, the differences between the two groups were compared using the Mann–Whitney *U* test, and the differences among the three groups were compared using the Kruskal–Wallis H test. The count data were expressed as several patients and constituent ratios, and the *χ*^2^ test was used to compare the constituent ratio between two or more groups. A *P* value <0.05 indicated a statistically significant difference.

RETRACTED

## 3. Results and Analysis

### 3.1. Statistical Description of Observation Indicators of 233 Patients with Thrombocytopenia

The average duration of rhTPO treatment in 233 patients with thrombocytopenia was 5.99 days, the average time to increase platelets was 5.27 days, the average delay of the next chemotherapy or chemoradiotherapy cycle was 4.98 days, the prolonged hospitalization due to platelet decline was 4.44 days and the average increased hospitalization cost due to platelet decline was 6932.45 RMB, as shown in Table 1.

### 3.2. Comparison of Baseline Conditions in Patients with Grade II, III, And IV Thrombocytopenia

No significant differences were found in terms of gender and age distribution of patients (*P* > 0.05). However, there was a statistically significant difference in “with or without concurrent chemoradiotherapy” of grade II, III, and IV thrombocytopenia (*F* = 6.069, *P* = 0.048). Further pairwise comparisons found that the difference in concurrent chemoradiotherapy between patients with grade II and III thrombocytopenia was statistically significant (*χ*^2^ = 5.781, *P* = 0.016), but those between patients with grade III and IV thrombocytopenia and between patients with grade II and IV thrombocytopenia were not statistically significant (*P* > 0.05), as shown in Table 2.

### 3.3. Comparison of Indicators in rhTPO Treatment of Grade II, III, And IV Thrombocytopenia

After patients with grade II, III, and IV thrombocytopenia were treated with rhTPO, significant differences were observed in the days of rhTPO treatment, time to increased platelets, delay of the next chemoradiotherapy cycle, prolonged hospitalization due to platelet decline, increased hospitalization costs due to platelet decline, and with or without platelet transfusion (*P* < 0.05). Further pairwise comparisons found that the days of rhTPO treatment, time to increased platelets, delay of the next chemoradiotherapy cycle, increased hospitalization costs due to platelet decline, and the proportion of patients who received platelet transfusion were significantly lower in patients with grade II thrombocytopenia than in those with grade III thrombocytopenia, and the differences were statistically significant (*P* < 0.05); the proportion of patients who received platelet transfusion after rhTPO treatment were significantly lower in patients with grade III thrombocytopenia than in those with grade IV thrombocytopenia, and the differences were statistically significant (*P* < 0.05); the days of rhTPO treatment, time to increased platelets, delay of the next chemoradiotherapy cycle, increased hospitalization costs due to platelet decline, and the proportion of patients who received platelet transfusion were significantly lower in patients with grade II thrombocytopenia than in those with grade IV thrombocytopenia, and the differences were also statistically significant (*P* < 0.05), as shown in Table 3.  Table 4 is the comparison of indicators in the use of rhTPO for the treatment of grade II and III thrombocytopenia.  Table 5 is the comparison of indicators in the use of rhTPO for the treatment of grade III and IV thrombocytopenia.  Table 6 is the comparison of indicators in the use of rhTPO for the treatment of grade II and IV thrombocytopenia.

RETRACTED

### 3.4. Economic Evaluation of rhTPO in the Treatment of Grade II, III, And IV Thrombocytopenia

As the severity of thrombocytopenia increased, all in costs, rhTPO treatment costs, platelet costs, drug costs, and nondrug costs also showed an upward trend, as shown in Figure 1. The results demonstrated that there are significant differences in whether or not concurrent chemoradiotherapy is used in patients with grade II, III, and IV thrombocytopenia. As the severity of thrombocytopenia increased, all in costs, rhTPO treatment costs, platelet costs, drug costs, and nondrug costs also showed an upward trend. rhTPO has good clinical efficacy in the treatment of chemotherapy- or chemoradiotherapy-induced thrombocytopenia. The economic evaluation of rhTPO in the treatment of grade II thrombocytopenia is positive.

## 4. Conclusion

In summary, when it comes to clinical treatment, a reasonable choice of treatment should be made according to the economic status and willingness of patients. The best treatment regimen with the best efficacy, safety, short course, and low cost should be done in the clinic as much as possible.

In this paper, the clinical efficacy and economic evaluation of recombinant human thrombopoietin (rhTPO) in the treatment of grade II, III, and IV thrombocytopenia induced by chemotherapy or chemoradiotherapy are investigated. Conclusively, rhTPO has good clinical efficacy in the treatment of chemotherapy- or chemoradiotherapy-induced thrombocytopenia. Patients with grade II, III, or IV thrombocytopenia should be treated as early as possible so that platelet levels can be restored as quickly as possible with a shorter treatment time and a lower cost. However, our study was conducted from a retrospective survey with a relatively small sample size in which all patients had been diagnosed with lung cancer at our hospital. Subsequent confirmation of the above is warranted by conducting multicenter studies with large samples. Reference [6], [9].

RETRACTED

## Figures and Tables

**Figure 1:** Economic evaluation of the use of rhTPO in patients with different grades of thrombocytopenia.

**Table 1:** Statistical description of observation indicators of 233 patients with thrombocytopenia.

Indicators	Mean ($\bar{x}$)	Standard deviation (s)	Median (M)	Upper and lower quartiles (P_25_, P_75_)	Minimum (min)	Maximum (max)
Age (years)	61.94	7.87	63.00	57.00, 67.00	26.00	79.00
Days of treatment	5.99	4.30	5.00	3.00, 7.50	1	40
Time to increase platelets (days)	5.27	3.88	4.00	3.00, 7.00	0	21
Delay of the next chemoradiotherapy cycle (days)	4.98	8.61	2.00	0,7.00	0	91
Prolonged hospitalization due to platelet decline (days)	4.44	7.35	3.00	0,7.00	0	91
Increased hospitalization costs due to platelet decline	6932.45	4790.42	6048.00	4032.00, 8566.00	1008.0	42120.0

**Table 2:** Comparison of baseline conditions in the use of rhTPO for treatment of grade II, III, and IV thrombocytopenia [*n*, (%)].

Characteristics	Use of recombinant human thrombopoietin (rhTPO)			*χ* ^2^/F value	*P* value
	Grade II (*n* = 100)	Grade III (*n* = 94)	Grade IV (*n* = 39)		
Gender					
Male	80 (80.0)	72 (76.6)	27 (69.2)	1.832	0.400
Female	20 (20.0)	22 (23.4)	12 (30.8)		
Age ($\bar{x}$ ± *s*, years)	60.66 ± 8.47	62.84 ± 7.33	63.03 ± 7.20	2.337	0.099
Concurrent chemoradiotherapy					
No	68 (68.0)	48 (51.1)	25 (64.1)	6.069	0.048
Yes	32 (32.0)	46 (48.9)	14 (35.9)		

**Table 3:** Comparison of indicators in the use of rhTPO for treatment of grade II, III, and IV thrombocytopenia [*n*, (%)].

Indicators	Use of recombinant human thrombopoietin (rhTPO)			*χ* ^2^ value	*P* Value
	Grade II (*n* = 100)	Grade III (*n* = 94)	Grade IV (*n* = 39)		
Delay of the next chemoradiotherapy/radiotherapy cycle due to platelet decline					
No	56 (56.0)	40 (42.6)	14 (35.9)	5.921	0.052
Yes	44 (44.0)	54 (57.4)	25 (64.1)		
Regimen change due to altered platelet count					
No	85 (85.0)	88 (93.6)	32 (82.1)	4.962	0.084
Yes	15 (15.0)	6 (6.4)	7 (17.9)		
Dose reduction of chemoradiotherapy due to platelet decline					
No	85 (85.0)	81 (86.2)	31 (79.5)	0.970	0.616
Yes	15 (15.0)	13 (13.8)	8 (20.5)		
Days of treatment	5.00 (3.00, 6.00)	6.00 (4.00, 8.00)	6.00 (4.00, 11.00)	16.319	<0.001
Time to increase platelets (days)	3.00 (2.00, 5.00)	5.50 (3.00, 8.00)	6.00 (3.00, 11.00)	31.828	<0.001
Delay of the next chemoradiotherapy cycle (days)	0 (0, 5.75)>	3.00 (0, 9.25)	3.00 (0, 8.00)	8.460	0.015
Prolonged hospitalization due to platelet decline (days)	1.00 (0, 6.00)	3.50 (0, 7.00)	5.00 (0, 8.00)	7.908	0.019
Increased hospitalization costs due to platelet decline	5040.00 (3024.00, 6979.00)	6503.00 (5040.00, 9474.00)	7440.00 (5874.00, 14410.00)	35.347	<0.001
Platelet transfusion					
No	95 (95.0)	67 (71.3)	16 (41.0)	47.616	<0.001
Yes	5 (5.0)	27 (28.7)	23 (59.0)		

RETRACTED

**Table 4:** Comparison of indicators in the use of rhTPO for treatment of grade II and III thrombocytopenia [*n*, (%)].

Indicators	Use of recombinant human thrombopoietin (rhTPO)		Z/*χ*^2^ value	*P* Value
	Grade II (*n* = 100)	Grade III (*n* = 94)		
Days of treatment	5.00 (3.00, 6.00)	6.00 (4.00, 8.00)	−3.610	<0.001
Time to increase platelets (days)	3.00 (2.00, 5.00)	5.50 (3.00, 8.00)	−4.977	<0.001
Delay of the next chemoradiotherapy cycle (days)	0 (0, 5.75)	3.00 (0, 9.25)	−2.602	0.009
Prolonged hospitalization due to platelet decline (days)	1.00 (0, 6.00)	3.50 (0, 7.00)	−1.821	0.069
Increased hospitalization costs due to platelet decline	5040.00 (3024.00, 6979.00)	6503.00 (5040.00, 9474.00)	−4.900	<0.001
Platelet transfusion				
No	95 (95.0)	67 (71.3)	19.798	<0.001
Yes	5 (5.0)	27 (28.7)		

**Table 5:** Comparison of indicators in the use of rhTPO for treatment of grade III and IV thrombocytopenia [*n*, (%)].

Indicators	Use of recombinant human thrombopoietin (rhTPO)		Z/*χ*^2^ value	*P* Value
	Grade III (*n* = 94)	Grade IV (*n* = 39)		
Days of treatment	6.00 (4.00, 8.00)	6.00 (4.00, 11.00)	−0.761	0.447
Time to increase platelets (days)	5.50 (3.00, 8.00)	6.00 (3.00, 11.00)	−1.023	0.306
Delay of the next chemoradiotherapy cycle (days)	3.00 (0, 9.25)	3.00 (0, 8.00)	−0.094	0.925
Prolonged hospitalization due to platelet decline (days)	3.50 (0, 7.00)	5.00 (0, 8.00)	−1.304	0.192
Increased hospitalization costs due to platelet decline	6503.00 (5040.00, 9474.00)	7440.00 (5874.00, 14410.00)	−1.871	0.061
Platelet transfusion				
No	67 (71.3)	16 (41.0)	10.752	0.001
Yes	27 (28.7)	23 (59.0)		

**Table 6:** Comparison of indicators in the use of rhTPO for treatment of grade II and IV thrombocytopenia [*n*, (%)].

Indicators	Use of recombinant human thrombopoietin (rhTPO)		z/*χ*^2^ value	*P* value
	Grade II (*n* = 100)	Grade IV (*n* = 39)		
Days of treatment	5.00 (3.00, 6.00)	6.00 (4.00, 11.00)	−2.955	0.003
Time to increase platelets (days)	3.00 (2.00, 5.00)	6.00 (3.00, 11.00)	−4.235	<0.001
Delay of the next chemoradiotherapy cycle (days)	0 (0, 5.75)	3.00 (0, 8.00)	−2.235	0.025
Prolonged hospitalization due to platelet decline (days)	1.00 (0,6.00)	5.00 (0,8.00)	−2.655	0.008
Increased hospitalization costs due to platelet decline	5040.00 (3024.00, 6979.00)	7440.00 (5874.00, 14410.00)	−4.755	<0.001
Platelet transfusion				
No	95 (95.0)	16 (41.0)	50.813	<0.001
Yes	5 (5.0)	23 (59.0)		

RETRACTED

## Data Availability

The simulation experiment data used to support the findings of this study are available from the corresponding author upon request.
